This article has been retracted.

# Lentinan Enhances the Function of Oxaliplatin on the Esophageal Tumors by Persuading Immunogenic Cell Death

**DOI:** 10.1155/2022/2296574

**Published:** 2022-07-08

**Authors:** Xiaolei Huo, Zhen Pei, Weiwei Wang, Yu Liu, Jing Sun, Hui Wang, Nanping Ai

**Affiliations:** ^1^Department of Basic Medicine, Changzhi Medical College, Changzhi, Shanxi Province, China; ^2^Changzhi Maternal and Child Health Care Hospital, Changzhi, Shanxi Province, China

## Abstract

**Objective:**

The focus of this research was to look at the effects of the combination of the lentinan (LNT) and oxaliplatin (Oxa) on the apoptosis of human esophageal cancer cells, as well as the underlying mechanism.

**Methods:**

LNT and Oxa were used to treat EC-109 human esophageal cancerous cells at various doses, and the cell survival rate was measured using the Cell Counting Kit-8 (CCK-8) assay. In addition, 24 h after treatment of EC-109 cells with a combination of LNT and Oxa, flow cytometry was used to analyze their apoptotic effect on these cells. Additionally, LNT on EC-109 cell apoptotic upshot was assessed via measuring the consequence of LNT on the mRNA and protein expression levels pertaining to immunogenic cell death factors CALR, HSP90, and HSP70 by qPCR (quantitative real-time polymerase chain reaction) and western blot analysis, correspondingly.

**Results:**

Cell proliferation was inhibited only when EC-109 cells were added with LNT at 1,200 *μ*g/mL to the maximum concentrations, but the combination of LNT and Oxa at a low dose (800 *μ*g/mL and 20 *μ*M, respectively) significantly increased their sensitivity to Oxa and reduced their proliferation (*P* < 0.05), and their apoptosis was significantly increased by LNT (*P* < 0.05). The immunogenic cell death-related genes CALR, HSP90, and HSP70 had dramatically enhanced mRNA and protein expression levels after therapy with a combination of LNT and Oxa (*P* < 0.05).

**Conclusion:**

These data imply that LNT increases the susceptibility of esophageal cancerous cells to Oxa by driving EC-109 cells to display immunogenic death. Therefore, LNT combined with Oxa may be an effective method in esophageal cancer management.

## 1. Introduction

Human tumor incidence and death have been steadily rising in recent years, and the incidence of esophageal cancer, in particular, remains high. Esophageal cancer is the sixth leading cause of cancer-related deaths of men, and the overall 5-year survival rate diverses from 15 to 25% worldwide [1]. Squamous cell carcinoma (SCC) and adenocarcinoma (AC) are two major subtypes of esophageal cancer.

The current main treatment technique for esophageal cancer is surgery, either alone or in conjunction with chemotherapy and/or radiotherapy, and the prevalence of esophageal malignancy has remained high in recent years [2, 3]. However, although surgical treatment and systemic chemotherapy can be used to treat esophageal cancer and prolong the patient survival to some degree, they cannot effectively treat advanced esophageal cancer. Currently, there are no effective drugs for esophageal cancer treatment except for those targeting PD-L1 in PD-L1-positive cancer [4, 5]. Oxaliplatin- (Oxa-) based chemotherapy regimens are still one of the main clinical regimens for esophageal cancer treatment, but the development of resistance to Oxa and its toxicity limits its efficacy in the treatment of esophageal cancer [6, 7]. Reducing its cytotoxicity and preventing the development of resistance to Oxa in esophageal cancer remains an unsolved challenge in the treatment of this cancer.

Extracts from natural foods and herbs for cancer treatment have received widespread attention from researchers due to their advantages of little side effects [8, 9]. Lentinan (LNT) is a polysaccharide compound derived from shiitake mushroom (Lentinula edodes) mycelium, thus exhibits therapeutic effects such as antioxidative stress, anti-inflammatory, and anticancer and has been widely used in cancer adjuvant therapy clinical trials [10–12]. Oxa is a commonly used platinum-based chemotherapeutic agent and is used in combination with other drugs. LNT in combination with paclitaxel or cisplatin efficiently inhibits gastric cancer cell growth and promotes apoptosis, and LNT in conjunction with cisplatin greatly minimises the adverse effects of cisplatin and can successfully enhance the standard of life of lung cancer patients. However, its role in esophageal cancer is currently unclear. In the current research, we appraised the antitumor immune outcome of LNT alone and with Oxa combination against esophageal cancer by determining the alteration of the apoptotic mechanism in esophageal cancer cells.

This study will demonstrate the role of lentinan and Oxa on the esophageal tumors and explain the underlying mechanism, which will bring light on the treatment of patients.

## 2. Results

### 2.1. Both LNT and Oxa Inhibit Proliferation and Induce Apoptosis in EC-109 Esophageal Tumor Cells

We cocultured EC-109 cells with different concentrations of LNT (0 1,600 g/mL) and Oxa (0 80 m) for 24 to 72 hours to test the impacts of LNT and Oxa on the proliferation of EC-109 esophageal cancer cells and then used the Cell Counting Kit-8 (CCK-8) assay to determine the growth inhibitory effects of LNT and Oxa on EC-109 cells. Both LNT (Figure 1(a)) and Oxa (Figure 1(b)) decreased the growth of EC-109 cells, and cytotoxicity was inversely linked with drug concentration and duration of treatment as measured by the cell value-added rate. The following formula was used to estimate cell viability:

(1) $$\begin{array}{c} \text{Cell viability}\left(\%\right)=\frac{\left(\text{ODtreated}-\text{ODbackground}\right)}{\text{ODunterated}-\text{ODbackground}}*100\% \end{array}$$

We used flow cytometry and an Annexin V-fluorescein isothiocyanate (FITC)/propidium iodide (PI) apoptosis assay to determine the rate of apoptosis of EC-109 cells after treatment with LNT for 48 hours to see if the inhibitory effect of LNT on EC-109 cell growth was related to its apoptosis-inducing effect. The apoptosis rate of EC-109 cells rose in a dose-dependent manner as the LNT concentration was increased, similar to the results of the CCK-8 experiment. These findings revealed that LNT induced apoptosis in EC-109 cells (*P* < 0.05) (Figure 2).

### 2.2. LNT Enhances the Sensitivity of EC-109 Cells to Oxa

The use of drug combinations in the therapeutic practice of malignancies is a frequent practice. The impacts of the conjunction of LNT and Oxa on the proliferation and apoptosis of EC-109 cells were assessed using the CCK-8 assay and flow cytometry to see if the combination of LNT and Oxa may increase the cell proliferation inhibition activity and apoptosis-inducing effect of Oxa on EC-109 cells. The outcomes explored it, and the TLN and Oxa combination significantly enhanced both the proliferation inhibitory effect and apoptosis-inducing effect of Oxa on EC-109 cells (Figures 3(a) and 3(b)).

Using qPCR and western blot analysis, we examined the mRNA and protein expression levels of BAX, Bcl-2, and caspase 3 in EC-109 cells to see if the combination of LNT and Oxa was linked with elevated mRNA and protein expression levels of genes involved in apoptotic pathways. The results demonstrate the effectiveness of LNT and Oxa in increased BAX and caspase 3 mRNA and protein expression (*P* < 0.01) while inhibiting Bcl-2 mRNA and protein expression (*P* < 0.05) (Figures 3(c) and 3(d)).

The combination index (CI) is one of the important measurement indexes to assess the degree of interaction between drugs. A CI < 1 denotes that there could be a synergistic impact between two medicines, a CI > 1 indicates that the relationship between 2 medicines is antagonistic, and a CI = 1 denotes the cumulative effect of the two drugs. To learn more about how the combination of LNT mechanism and Oxa to determine whether it was a cumulative or synergistic effect mechanism, we analyzed the combination index (CI) using the CompuSyn software. The results showed that the CI was <1, implying that Oxa and LNT's combined action on EC-109 cells was primarily synergistic (Figure 3(e)).

### 2.3. LNT Augments the Sensitivity of the EC-109 Cells to Oxa by Activating the Immunogenic Cell Death Pathway in EC-109 Cells

Immunogenic cell death (ICD), a type of controlled cell death, is linked to DAMPs (damage-associated molecular patterns), which occur when antigens are released intracellularly and cause self-damage in cells [13]. It has been shown that LNT can promote H22 cell death by inducing the expression of more CALR, HMG1, and HSP70 on the surface of H22 cells. We further investigated how LNT, in combination treatment with Oxa, enhances Oxa-induced apoptosis in EC-109 cells using ELISA, analysis of qRT-PCR, and western blot analysis to measure levels of key molecules associated with ICD and ATP, in addition to flow cytometry to assess the expression of surface (cell) immune antigens on EC-109 cells. The results of the ELISA of supernatants showed significantly higher release of CXCL10 and IL17 (*P* < 0.05) and significantly upregulated levels of HSP90 and HSP70 (*P* < 0.05) in the supernatants of the LNT and Oxa+LNT groups related to control. The relative mRNA expression levels of HMGB1, CALR, ANXA1, and IFNA1 were considerably greater (*P* < 0.05), while the relative protein expression levels of HSP70, HSP90, and CALR were dramatically increased, according to the results of the qRT-PCR and western blot studies (*P* < 0.05). These results indicated that LNT can enhance the toxicity of Oxa to cells by activating the release of ICD proteins in EC-109 cells (Figure 4).

## 3. Materials and Methods

### 3.1. Cell Culture

The human esophageal melanoma EC-109 cells (Shanghai Cell Bank of the Chinese Academy of Sciences, Shanghai, China) have been cultured in RPMI-1640 complete medium (Invitrogen, Carlsbad, CA, USA) containing 100 U/mL penicillin and streptomycin (Invitrogen) and 10% foetal bovine serum (Invitrogen) at 37°C in an incubator with 5% CO_2_.

### 3.2. CCK-8 Assay

The Cell Counting Kit-8 (CCK-8) test (Beyotime Biotechnology, Shanghai, China) was used to calculate the cell survival rate. EC-109 cells in the logarithmic growth phase were collected and planted at a density of 5,000 cells per well in 96-well plates, and afterwards, the cells were attached and grown to 60% confluence, and each plate was incubated for 24 or 48 h with the corresponding concentration of the drug. The plate was then incubated at 37°C for 1-4 hours after 10 mL of CCK-8 solution was introduced to each well. The cell survival rate percent was then estimated for each group by detecting the optical density value at 450 nm (OD450), as follows: cell survival rate% = (OD_450_ value of drug group − OD_450_ of blank wells)/(OD_450_ of the control group − OD_450_ of the blank group) × 100%.

### 3.3. Analysis of Drug Synergy Using the CompuSyn Software

Based on the findings of the CCK-8 test, OD_450_ value and survival rate percentage at each drug concentration were obtained and analyzed with the CompuSyn software [ComboSyn Inc., Paramus, (NJ), 2005. http://www.combosyn.com [Donated to biomedical communities for free download, upon registration, beginning August 1. 2012 via http://www.combosyn.com of PD Science LLC].]. If CI < 1, the drug has synergistic effect, and the smaller the value, the more significant the synergistic effect; if CI = 1, it means that the drug has a cumulative effect; if CI > 1, it means that the drug has an antagonistic effect, and the value The larger the value, the more significant the antagonistic effect.

### 3.4. Apoptosis Assay

To determine the manner of cell death, researchers employed an Annexin V-fluorescein isothiocyanate (FITC)/propidium iodide (PI) apoptosis detection kit (Keygentec, Nanjing, China) (apoptosis versus necrosis). As mentioned in Collect cells as in step 2.2, log-phase grown EC-109 cells were harvested, plated in 96-well plates, and treated with the appropriate drug dose. Flow cytometry was used to examine EC-109 cells in the logarithmic growth phase for apoptosis using the Annexin V-FITC/PI double-staining method. The cells from each group were collected, centrifuged at 1,000*g* for 35 minutes, washed twice with precooled phosphate-buffered saline (PBS), and finally resuspended at a concentration of 1 × 10^6^/mL.

The cell suspension was then mixed with 250 mL of diluted binding buffer, and 100 mL of the mixture was put into a 5 mL flow cytometry tube. The cell suspension was blended well and incubated for 15 minutes at ambient temp in the dark after adding 5 *μ*L of Annexin V-FITC and 10 *μ*L of 20 g/mL PI solution. The cell suspension was then examined using flow cytometry after 400 L PBS was added to the reaction tube.

### 3.5. Quantification of Secreted ATP, IL-17, CXCL10, HSP70, and HSP90

After 48 hours of incubation with 800 g/mL LNT or 20 M Oxa, the supernatant was collected, and the cell pellet was discarded after centrifugation (15,000 rpm, 30 min). Western blot analysis and enzyme-linked immunosorbent assays were used to evaluate the quantities of IL17, CXCL10, HSP70, and HSP90 released into the supernatant (ELISA). According to the manufacturer's instructions, the total protein content in the supernatant was determined using the Pierce bicinchoninic acid (BCA) Protein Assay Kit (Thermo Fisher Scientific Inc., Waltham, MA, USA). Following the determination of the total protein content in the supernatant, aliquots of 20-30 g of protein were combined with loading buffer, boiled in a boiling water bath for 5 minutes, and chilled to room temperature. The proteins in the aliquots were then separated on 10 percent SDS-PAGE gels and transferred to PVDF membranes using sodium dodecyl sulfate-polyacrylamide gel electrophoresis (SDS-PAGE). The membranes were then blocked for 1 hour at room temperature with 5% fat-free dried milk in Tris-buffered saline (TBS) containing 0.1 percent Tween-20 (TBST), followed by overnight incubation with a primary antibody specific for HMGB1 (1 : 1,000, Sigma-Aldrich, Burlington, MA, USA). After that, the membranes were washed and incubated with a secondary antibody conjugated to horseradish peroxidase (1 : 2,000, MilliporeSigma) (HRP). The reference protein was bovine serum albumin (BSA). In addition, the levels of IL17, CXCL10, HSP70, and HSP90 in the collected supernatant were determined according to the manufacturer's instructions using IL17, CXCL10, HSP70, and HSP90 ELISA kits (Clonecloud, Wuhan, China). A chemiluminescent ATP determination kit was used to determine the amount of ATP in the collected supernatants (A22066, Invitrogen, Shanghai, China). The fluorescence decay was measured using a luminometer after separately mixing each collected supernatant with the chemiluminescent ATP determination kit reagent (containing the reaction mixture of the luciferin and firefly luciferase without ATP). A series of ATP standard curves were developed with varied ATP concentrations to determine the quantity of ATP in the supernatant.

### 3.6. Quantitative Real-Time Polymerase Chain Reaction (qPCR) Analysis

TRIzol reagent (Invitrogen) was used to extract total RNA from cells in different treatments according to the manufacturer's instructions. The whole RNA was then utilised to convert mRNA to cDNA using a reverse transcription kit (Promega Corporation, Madison, WI, USA; Cat# A2801). The relative expression levels of *BAX*, *BCL2*, *CASP3*, CALR, *HSP90*, and *HSP70* in EC-109 cells were measured by qPCR analysis with a qPCR Master Mix kit (Cat# A6000; Promega Corporation), using *GAPDH* as the internal reference. The 2-△△^ct^ method was utilized to compute the relative mRNA expression levels.

### 3.7. Western Blot Analysis

The concentration of the extracted protein was measured using the BCA Protein Assay Kit after total protein was extracted from EC-109 cells in the three treatment groups according to the kit instructions (Thermo Fisher Scientific Inc.). SDS-PAGE was used to separate the proteins, which were subsequently transferred to PVDF membranes as described in section. Western blot analysis with the following antibodies was used to evaluate the protein expression levels of BAX, BCL2, caspase 3,CALR, HSP90, and HSP70: anti-BAX (Cat# ab3191; Abcam, Cambridge, UK), anti-BCL2 (Cat# ab196495; Abcam), anti-Caspase 3 (Cat# ab179517, Abcam), anti-HSP90 (Cat# ab203085, Abcam), and anti-HSP70 (Cat# ab2787, Abcam). The western blot analysis was performed utilizing anti-GAPDH (Cat# ab8227; Abcam) as the internal reference protein.

### 3.8. Statistical Analysis

Data from three independent studies are provided as mean standard deviation. A one-way ANOVA was used to find differences between groups during statistical analysis. All analyses were carried out using IBMSPSS Statistics 21.0. A difference of *P* < 0.05 was considered statistically significant.

## 4. Discussion

Human tumor incidence and death have been steadily rising in recent years, and the incidence of esophageal cancer, in particular, remains high. One of the main reasons for tumor recurrence or difficulty in treatment is the weak immunogenicity or lack of expression of tumor antigens, and the body's immune tolerance to the tumor can lead to escape response when the tumor is attacked by the body, resulting in treatment failure [14–18]. Therefore, reducing tumor drug resistance and improving tumor immunogenicity is the key to successful esophageal tumor treatment.

An increasing number of natural immunogenic enhancing substances are receiving more and more attention from researchers. The combination of conventional chemotherapeutic or radiotherapeutic drugs with extracts from natural plants is used to reduce the resistance of chemotherapeutic or radiotherapeutic drugs to tumors while at the same time increasing the effective rate of action of chemotherapeutic or radiotherapeutic drugs [19–23]. Currently, natural plant extracts are considered effective substances to enhance drug efficacy and reduce toxicity and are widely used in a variety of cancers. The polysaccharide complexes extracted from natural shiitake mushrooms have been widely used in clinical practice. LNTs have been shown to have antioxidant, tumor-metastatic, tumor-proliferative, and immunomodulatory activities in vivo [24, 25]. However, the specific mechanism of its tumor-inhibitory activity is unclear. This work investigated the in vitro increase of the cellular level tumor suppression impact of LNT in conjunction with Oxa by activating ICD in esophageal cancer cells to elucidate the particular mode of action of LNT in esophageal cancer inhibition following treatment with Oxa.

Numerous studies have shown that LNT and Oxa can significantly inhibit tumor proliferation, metastasis, and invasion. LNT has been reported to inhibit SHG-44 human glioma cells [26], MCF-7 human breast cancer cell, and HepG2 human hepatocellular carcinoma cell [27] to varying degrees and can be used as an adjuvant in combination with chemotherapeutic agents to exert tumor-suppressive effects [28]. Oxa is a commonly used platinum-based chemotherapeutic agent and is used in combination with other drugs. LNT in combination with paclitaxel or cisplatin efficiently inhibits gastric cancer cell growth and promotes apoptosis, and LNT in conjunction with cisplatin greatly minimises the adverse effects of cisplatin and can successfully enhance the standard of life of lung cancer patients. Zhang et al. demonstrated [10] that LNT can regulate autophagy and apoptosis to inhibit the development of rectal cancer. The combination of LNT and Oxa was found to have significant synergistic antitumor effects in H22-bearing mice and effectively reduced the toxic side effects caused by Oxa. The antiproliferative effects of LNT and Oxa on EC-109 cells were time and dose dependent, according to the findings. The combination group significantly showed inhibited cell proliferation compared with LNT or Oxa alone. Moreover, CI analysis with the CompuSyn software also indicated the synergistic antiproliferative effects of LNT in combination with Oxa. Flow cytometric analysis revealed that the EC-109 cell apoptosis was significantly higher posttherapy in a combination of LNT and Oxa than with Oxa alone (*P* < 0.05), implying that the two medicines combined may suppress cell proliferation by increasing cell sensitivity to Oxa.

ICD is a distinct type of controlled cell death, thus related to DAMPs associated with the release of antigens from cells leading to the production of self-damage in tumor cells [13]. Antigenic molecules released from the cell surface area are among the important markers of ICD, including ATP, HMGB1, HSP90, and HSP70. Natural plant extracts have been demonstrated to be effective in a number of investigations with the ability to induce an increase in the secretion of ATP, HSP90, and HSP70 from tumor cells which can more effectively inhibit tumor growth, proliferation, and metastasis. W. Wang et al. [29] showed that LNT can promote H22 cell death by inducing the expression of CALR, HMG1, and HSP70 on the surface of H22 cells. Similar results were obtained in this study, in which a significantly increased level of CALR was found in the culture supernatant of LNT-treated EC-109 cells, suggesting that CALR is transferred from inside the cells to the cell surface, which in turn promotes ICD in EC-109 cells. Oxa was not found to have a role in promoting ICD in Oxa-treated EC-109 cells. The combination of LNT and Oxa was found to induce the release of ATP, CALR, HSP70, and Hsp90 from EC-109 cells, which increased the cell death of EC-109 cells.

The advantage of this study was that this study demonstrated the role of LNT in assisting the function of Oxa in esophageal tumor cells, which will bring light for patients. However, there are also limits of this study. The mechanism was not clearly clarified and needs further studies deeply.

## 5. Conclusion

The results of this study showed that treatment of EC-109 cells with a combination of LNT and Oxa significantly increased their level of ATP and their release of CALR and other immunogenic signaling substances related to apoptosis, which increased the rate of apoptosis while at the same time increasing autoimmunogenicity. In future studies, we will analyze the ICD process in EC-109 cells induced by LNT combined with oxaliplatin and its specific mechanisms of action and pathways.

## Figures and Tables

**Figure 1:** Both LNT and Oxa showed growth inhibitory effects against EC-109 cells. The vitality of EC-109 cells was measured using the CCK-8 assay after they were exposed to various amounts of LNT or Oxa for 24 to 72 hours. Each experiment was repeated three times, with the findings given as the mean minus the standard deviation.  ^∗^24 h compared with 48 h and 72 h, *P* < 0.05.

**Figure 2:** LNT induces apoptosis of EC-109 cells. (a–e) Rate of EC-109 cells apoptosis under the action of different concentrations of LNT. (f) Apoptosis rate of cells; each experiment was repeated 3 times, uttered like mean ± standard deviation. ^∗^*P* < 0.05 vs. 0*μ*g/mL LNT. Differences between groups have been detected by statistical analysis of one-way variance.

**Figure 3:** LNT enhances the sensitivity of EC-109 cells to Oxa. (a) The conjunction of LNT and Oxa greatly reduced EC-109 cell growth (*P* < 0.05). (b) The combination of LNT and Oxa persuaded programmed cell death in EC-109 cells (*P* < 0.05). (c) LNT combination and Oxa induced mRNA expression levels of *BAX* and *CASP3* and inhibited the mRNA expression *BCL2* (*P* < 0.05) level. (d) The conjunction of LNT and Oxa increased BAX and cleaved caspase 3 protein expression while suppressing BCL2 protein expression (*P* 0.05). (e) The analysis of the combination index (CI) of LNT and Oxa using the CompuSyn software revealed that both LNT and Oxa acted synergistically on EC-109 cells. The data were expressed as the mean standard deviation for each experiment, which was done in triplicate. *P* < 0.05 in comparison to 0 g to analyze the differences between groups; statistical analysis using one-way analysis of variance (ANOVA) was used.

**Figure 4:** LNT-induced immunogenic cell death (ICD) pathway in EC-109 cells enhances the effectiveness of the combined Oxa intervention. (a) LNT alone or combined with Oxa induced the release of ATP, CXCL10, IL17, HSP70, and HSP90 (*P* < 0.05). (b) LNT alone or combined with Oxa induced the mRNA expression levels of *HMGB1*, *ANXA1*, *IFNA1*, and *CALR* (*P* < 0.05). (c) CALR, HSP70, and HSP90 protein expression levels were increased by LNT alone or in combination with Oxa (*P* < 0.05). Each experiment was repeated three times, with the findings given as mean ± standard deviation. ^∗^Contrast with control at *P* < 0.05. To find differences between the groups, statistical analysis using one-way analysis of variance (ANOVA) was used.

## Data Availability

The data used to support this study is available from the corresponding author upon request.
